The article "Prognostic Value of Histidine-Rich Glycoprotein for Community-Acquired Pneumonia" was published in 2022. Journal: Dis Markers.

# Prognostic Value of Histidine-Rich Glycoprotein for Community-Acquired Pneumonia

**DOI:** 10.1155/2022/4713045

**Published:** 2022-02-01

**Authors:** Xinwei He, Qiongzhen Luo, Lili Zhao, Ying Shang, Zhancheng Gao

**Affiliations:** ^1^Department of Internal Medicine, Xicheng District Zhanlanlu Hospital, Beijing, China; ^2^Department of Respiratory & Critical Care Medicine, Beijing Tsinghua Changgung Hospital, School of Clinical Medicine, Tsinghua University, Beijing, China; ^3^Department of Respiratory & Critical Care Medicine, Peking University People's Hospital, Beijing, China

## Abstract

**Purpose:**

Histidine-rich glycoprotein (HRG) is abundant in serum and has been implicated in several processes including blood coagulation and immune response. This prospective study is aimed at exploring HRG as a biomarker in patients hospitalized for community-acquired pneumonia (CAP).

**Methods:**

A total of 160 patients (73 severe CAP, 57 nonsevere CAP), and 30 healthy controls were enrolled in 2019. Demographic and clinical data were recorded for all patients. Serum HRG concentration was measured upon admission using ELISA.

**Results:**

HRG levels were significantly lower in severe CAP patients compared with other groups, regardless of etiology, and were negatively correlated with serum interleukin-6 and disease severity index scores. Combination of CURB-65, PSI, and APACHE II scores with HRG values significantly improved the accuracy of predicting 30-day mortality in these patients. Cox regression analysis showed that HRG could serve as an independent risk factor for 30-day mortality. Notably, patients with HRG ≤ 16.92 *μ*g/mL had significantly lower cumulative survival than those with HRG > 16.92 *μ*g/mL.

**Conclusion:**

Serum HRG levels are lower in patients with severe CAP and are negatively correlated with disease severity scores. Measurement of HRG upon admission can provide valuable prognostic information for patients with CAP.

## 1. Introduction

Community-acquired pneumonia (CAP) poses a major threat to public health as a high morbidity and high mortality infectious disease [1]. Due to the complexity of its etiology and pathogenesis, CAP prognosis can be extremely variable, ranging from mild to fatal. Accurate prediction of CAP severity and subsequent prognosis can promote the development of timely and effective treatment strategies. Thus, several clinical measures have been established to assess CAP disease severity, including scoring systems and biomarkers. The most commonly used scoring indexes include CURB-65 (confusion, uremia, respiratory rate, blood pressure, and age ≥ 65 years) [2] and the pneumonia severity index (PSI) [3]. However, CURB-65 incorporates only a limited number of factors specific CAP, while the PSI system relies more heavily on age and underlying pathologies. To address this issue, several biomarkers have been widely examined for their ability to determine severity or provide reliable prognosis to help resolve pneumonia-related clinical uncertainties.

Recent studies have reported that histidine-rich glycoprotein (HRG), also called histidine-proline-rich glycoprotein, levels are lower in cases of systemic inflammatory response syndrome (SIRS) [4] or among patients with ventilator-associated pneumonia (VAP) [5], and that these levels were significantly correlated with prognosis. These results indicate that HRG may be a promising candidate biomarker for CAP infection. HRG is an abundant and multimodular serum glycoprotein that is mainly produced in the liver but can also be synthesized by monocytes and macrophages [6]. HRG binds to various ligands, including plasminogen, fibrinogen, and phospholipids, thereby contributing to blood coagulation and fibrinolysis [7], immune response [8], and tumorigenesis [9], among other processes. In particular, HRG has been reported to modulate phagocytosis and to exhibit antibacterial activity *in vitro* [10]. Additionally, mice lacking HRG were found to be more susceptible to bacterial [11] and fungal [12] infections.

Based on these previous findings, we hypothesized that the HRG levels detected upon admission could have prognostic value for patients with CAP. Here, in this work, we prospectively evaluated HRG levels in a cohort of patients with CAP to clarify whether patients with different severities of CAP exhibited differences in HRG levels, thus, indicating potential clinical significance.

## 2. Materials and Methods

### 2.1. Study Design

The study was conducted at Peking University People's Hospital, Beijing Xicheng District, Zhanlanlu Hospital, China, during the period of January through December 2019. Consecutive adult patients (age > 18 years) diagnosed with CAP were recruited within 8 h of their admittance CAP was defined according to (1) disease onset in the community; (2) the presence of respiratory symptoms, such as cough and sputum production, or signs of inflammation (including fever and elevated white blood cell (WBC) count); (3) presentation with newly emerging changes in chest imaging [13]. Pregnant women, patients with immunosuppressive conditions, or diagnosis other than CAP were excluded from the study. A total of 30 healthy volunteers (age > 18 years) were enrolled as a control group. This study was approved by the Medical Ethics Committee of Peking University People's Hospital.

For this study, we based our diagnosis of severe CAP on observations of a minimum of one major criterion or three minor criteria, as described in previous studies [14]. Major criteria: (1) mechanical ventilation was administered, and (2) vasopressors were applied for patients who experienced septic shock. Minor criteria: (1) patient presented with a respiratory rate ≥ 30 breaths/min; (2) oxygenation index (PaO_2_/FiO_2_) ≤ 250; (3) multilobar infiltrates were observed through radiography; (4) patient exhibited disorientation or appeared confused; (5) serum levels of urea nitrogen were ≥20 mg/dL; (6) WBC counts were ≤4 × 109; (7) platelet counts < 100 × 109/L; (8) patient's core body temperature was lower than 36.0°C; and/or (9) patient displayed hypotension which required aggressive fluid resuscitation. The primary endpoints of the study were hospital mortality and discharge.

### 2.2. Data Collection

Demographic data and clinical history were recorded for each patient upon hospital admission. Documented information included patient age, sex, smoking habits, comorbidities, and pretreatment with antibiotics in the five days preceding admission. In the first 24 hours of hospital stay, patients were also tested for WBC count, c-reactive protein (CRP) levels, procalcitonin (PCT) levels, blood biochemistry, and thoracic imaging. Based on the recorded data and thorough examination, index scores for CURB-65, PSI, and acute physiology and chronic health evaluation (APACHE) II were determined for each patient. All patients were treated individually in accordance with Chinese antibiotic guidelines [15].

To detect HRG, we obtained venous blood samples from each patient in the first 8 h following admission. Samples were collected and centrifuged in sterile, and procoagulation tubes and the serum were stored in a −80°C freezer for later analysis. Patients with low quantity or low quality serum samples were consequently excluded from the study.

### 2.3. Measurement of HRG and Interleukin-6 Levels

Enzyme-linked immunosorbent assay (ELISA) kits (ELH-HPRG, RayBiotech Life, Norcross, GA, USA) were used to quantify serum levels of HRG in duplicate, following the protocols provided with the kit. A standard spectrophotometer (Multiskan FC, Thermo Fisher Scientific, Waltham, MA, USA) was used to determine light absorbance at 450 nm (A450). The lower limit of detection was found to be 1.23 ng/mL, while inter- and intra-assay coefficients of variation were <12%. Serum interleukin- (IL-) 6 was also quantified with ELISA kits (D6050, R&D Systems, Minneapolis, MN, USA), measured in duplicate for each sample, following the standard protocols for the kit. A Multiskan FC was used to determine A450, with correction at 570 nm. Standard curves for both HRG and IL-6 in serum were generated with CurveExpert Professional 2.6.3 (Hyams Development, Madison, WI, USA).

### 2.4. Statistical Analysis

For continuous variables with skewed data distribution, we calculated the median and interquartile range, while categorical variables were expressed as percentages. The Mann–Whitney *U* test was used to identify significant differences between two groups, and one-way analysis of variance and Kruskal-Wallis tests were applied for comparisons of three or more groups. In addition, Spearman's rho test was used to identify correlations between abnormally distributed variables. Thirty-day mortality was predicted for each patient using receiver operating curves (ROC). The impacts on 30-day survival rate by clinical variables were determined by Cox proportional hazards regression analysis, while Cox cumulative survival analysis tested whether HRG levels had independent effects on 30-day mortality. Statistical tests were two-sided, with significance determined at *p* < 0.05. SPSS (v20.0; IBM Corp, Armonk, NY, USA) and Prism 7 (GraphPad Software, San Diego, CA, USA) were used to perform all statistical tests.

## 3. Results

### 3.1. Patient Characteristics

In total, 160 patients were enrolled in this study (median age: 56 years; interquartile range: 37–68 years). A full list of baseline characteristics for all patients is shown in Table 1. Overall, 74 (46.3%) patients were diagnosed with severe CAP, among whom 28 were diagnosed within 48 h of hospital admission and 46 developed severe CAP after a median of 4 days following admission. Eleven (6.9%) patients died during hospitalization within 11–26 days, and two patients died after more than 30 days of hospitalization. The main cause of death was confirmed to be rapid progression of CAP or its complications, including seven patients who died due to septic shock and six patients who died of multiple organ failure.

Among this cohort, 140 (87.5%) patients were discharged with improved health conditions within 30 days (median: 12 days; range: 9–17 days), and seven (4.4%) patients were discharged after more than 30 days of hospitalization (range: 31–46 days).

### 3.2. HRG Levels and Etiology

Comparison of HRG levels showed no significant differences between healthy individuals and patients with nonsevere CAP (91.31 [74.75–102.00] vs. 75.37 [23.91–115.40] *μ*g/mL, respectively, *p* = 0.205), whereas HRG was significantly lower in patients with severe CAP (20.97 [8.58–75.97] *μ*g/mL, *p* < 0.001) compared with that of healthy individuals or patients with nonsevere CAP (Figure 1(a)).  Figure 1(b) showed that when patients with CAP were grouped by prognoses, HRG level was lowest in nonsurvivors (9.61 [6.91-13.37] *μ*g/mL, *p* < 0.001) compared with that of healthy individuals or survivors (62.57 [15.82-106.90] *μ*g/mL). While there was no significant difference in HRG levels among CAP patients when grouped by days of hospitalization (0-7 days, 8-14 days, 15-30 days, and ≥31 days) (Figure 1(c)).

In order to investigate whether HRG levels were associated with CAP etiology, we categorized CAP patients based on infection with bacteria, viruses, atypical pathogens (*Legionella pneumonia*, *Mycoplasma pneumonia*, and *Chlamydial pneumonia*), mixed pathogens, or unknown pathogens. We subsequently found that 41 (25.6%) patients had bacterial infection, 16 (10.0%) patients had viral infection, 12 (7.5%) patients were diagnosed with infection by atypical pathogens, 15 (9.4%) patients were infected with mixed pathogens, and 76 (47.5%) patients were infected by unknown pathogens. These patients had median HRG levels of 43.77 (9.63–109.20), 20.14 (8.30–62.23), 93.70 (62.35–113.70), 67.67 (36.17–114.60), and 42.12 (10.98–103.10) *μ*g/mL, respectively. No significant differences in HRG levels were found among any of the different etiology groups (*p* = 0.101) (Figure 1(d)).

### 3.3. Correlations between HRG Levels and CAP Severity

Comparison of HRG levels with CURB-65, PSI, and APACHE II indexes for CAP severity showed that among 160 patients with CAP, serum HRG concentration was negatively correlated with score values for all three systems (CURB-65 *r* = −0.356, PSI *r* = −0.357, and APACHE II *r* = −0.308; *p* < 0.001 in each test). Additionally, HRG levels showed a significant inverse correlation with IL-6 concentration (*r* = −0.359, *p* < 0.001) (Figure 2).

### 3.4. HRG Values in Predicting Prognosis in Patients with CAP

We next investigated whether HRG levels could be used to predict 30-day mortality in cases of severe CAP, summarized in Table 2. Analysis of area under the curve (AUC) for the ROC based on HRG levels was 0.810 (*p* < 0.001), and the optimal threshold HRG concentration for a prognosis of death was 16.92 *μ*g/mL (100% sensitivity, 72.79% specificity). Although the AUC for HRG was slightly less than that of CURB-65, PSI, and APACHE II (0.813, 0.874, and 0.923, respectively; Figure 3(a)), combining HRG concentration with these scores greatly improved the overall accuracy of prediction from 0.813 to 0.885 for CURB-65, 0.873 to 0.910 for PSI, and 0.923 to 0.947 for APACHE II (Figure 3(b)). Furthermore, Cox proportional regression analysis of the effects of HRG content on 30-day mortality rates for severe CAP patients revealed that only IL-6 (hazard ratio (HR) = 1.001; *p* = 0.001), HRG (HR = 0.889; *p* = 0.049), and APACHE II (HR = 2.020; *p* = 0.001) could serve as independent predictors of 30-day mortality risk, adjusted for clinical data (Table 3). Moreover, categorization of CAP patients based on high (>16.92 *μ*g/mL) or low serum HRG (≤16.92 *μ*g/mL) and subsequent analysis by Cox survival curves revealed that the low HRG group displayed significantly greater mortality rates than that of the high HRG group (*p* < 0.001, Figure 4), which was independent of other clinical parameters (i.e., age, bilateral lung infection, PCT, CURB-65, PSI, and APACHE II).

## 4. Discussion

This study revealed three major points: (1) HRG concentrations are significantly lower among severe CAP patients, regardless of etiology; (2) serum HRG content is inversely correlated with IL-6 levels and CURB-65, PSI, and APACHE II severity indexes; and (3) low serum HRG accumulation is an independent risk factor for 30-day mortality in patients with CAP. Collectively, our results indicate that low serum HRG is correlated with higher symptom severity and poor prognosis for CAP patients.

Previous reports have shown an association between low HRG levels and various diseases. For example, Winiarska et al. [16] found that serum HRG levels were decreased in patients with advanced lung cancer, and that specific concentrations were associated with late stages of lung cancer stage and hypofibrinolysis. Similarly, Ernst et al. [17] reported that plasma levels of HRG were significantly lower in patients with idiopathic pulmonary fibrosis (IPF) compared with those in healthy controls, but were positively correlated with values for forced vital capacity in these patients. Using a mouse model for acute pancreatitis, Terao et al. [18] found that decreased plasma HRG was associated with disease. In rheumatoid arthritis (RA), Kim et al. [19] reported that HRG was lower in patients with elevated levels of rheumatoid factor (RF), and that HRG levels could be used to distinguish patients with RA from healthy subjects (AUC = 0.861). In the present study, our results showed that HRG levels were significantly reduced in severe CAP patients, which is in agreement with previous studies that showed decreased HRG accompanies sepsis [4] and VAP [5]. Taken together, these studies indicate that HRG is a nonspecific biomarker in various pathological states.

In light of our finding that HRG was significantly reduced in cases of severe CAP, we further evaluated potential correlations between HRG levels and disease severity scores. These analyses revealed that low HRG concentrations are negatively correlated with CURB-65, PSI, and APACHE II, as well as with IL-6 values. IL-6 is widely used as a nonspecific indicator of immediate inflammatory response to infection. Several studies have reported that IL-6 could function as an informative or reliable predictor for determining the likelihood of treatment failure or mortality [20, 21]. Hence, these results also suggest that serum HRG could similarly aid in the clinical diagnosis of disease severity.

To the best of our knowledge, few studies have evaluated the effectiveness of HRG as a prognostic indicator. Kuroda et al. [4] previously reported that in 70 patients with SIRS, HRG level on day 1 of hospitalization was an independent prognostic factor after adjusting to APACHE II scores, with a cut-off value of 16.0 *μ*g/mL, and that mortality of the low HRG group was significantly higher than that of the high HRG group. Ding et al. [5] examined the serum HRG levels in 116 patients with VAP and found that serum HRG ≥ 29.5 *μ*g/mL was associated with a significantly higher rate of survival than HRG levels < 29.5 *μ*g/mL. In line with these findings, our study showed that HRG levels could enable the successful prediction of 30-day mortality in patients with CAP (AUC = 0.810). Although the predictive reliability of HRG was lower than that of CURB-65, PSI, and APACHE II, the predictive capacity for 30-day mortality of these severity indexes was significantly enhanced by integrating them with serum HRG values. Furthermore, consistent with other studies [4, 5], our results support that HRG can serve as an independent predictive marker for 30-day mortality among CAP patients. Additionally, when patients were grouped according to serum HRG concentrations higher or lower than 16.92 *μ*g/mL, the patients with high HRG were found to have a significantly higher survival rate than those with low HRG. Variation in this threshold between high and low values among studies could be related to differences in sample size or it may be specific to different diseases.

Several studies have investigated the functions of HRG during infection. Wake et al. [22] reported that knockdown of HRG exacerbated mortality in septic mice, and that therapeutic supplementation with HRG could improve survival. This effect may be related to inhibition of systemic inflammation and immunothrombosis, potentially through maintaining quiescence in circulating neutrophils and by controlling vascular endothelial cell activation. Furthermore, Gao et al. [23] studied microvascular breakdown during sepsis and found that HRG can preserve endothelial integrity via suppression of MAPK phosphorylation and Rho activation. It is thus reasonable to speculate that reduced serum HRG in sepsis or severe CAP could be due to its uptake by cells, which in turn worsens the disease manifestations. In addition, serum HRG levels were not correlated with CAP etiology, that is, unrelated to specific causative pathogens, which suggests that HRG could have multiple functions and can bind various ligands.

This prospective study had several limitations. First, HRG levels were only assessed during admission; therefore, the trends and response to treatment were not investigated. Second, among patients in each group of non-SCAP, SCAP, and survivors, serum HRG levels were quite discrete. It remains to be further studied whether HRG levels of some mild patients are temporarily increased or stress-induced. Third, there was no additional validation cohort to further support the present findings. A larger, multicenter study is necessary to confirm our results. Lastly, HRG, as a novel biomarker for severe CAP, should be compared with other reported markers, such as progranulin [24], midregional proadrenomedullin [25], soluble urokinase-type plasminogen activator receptor [26], or angiopoietin-1/2 [27]. Moreover, long-term prognostic information is limited since this study only investigated the predictive value of HRG for 30-day mortality. To date, no research has explored the predictive value of HRG for long-term prognosis.

In conclusion, serum HRG levels are significantly decreased in patients with severe CAP, independent of causative pathogen etiology. Low HRG serum levels are significantly associated with disease severity scores and, moreover, can enhance prognostic accuracy when these values are combined. Collectively, HRG assessment upon hospital admission may provide valuable prognostic information and help to rapidly diagnose patients with severe community-acquired pneumonia.

## Figures and Tables

**Figure 1:** Levels of histidine-rich glycoprotein (HRG) across multiple groups. (a) Levels of HRG in patients with community-acquired pneumonia (CAP) and healthy volunteers. In CAP patients, nonsevere vs. severe CAP, *p* < 0.001; non-CAP patients vs. healthy volunteers, *p* = 0.205. (b) Levels of HRG in healthy volunteers and CAP patients grouped by prognoses. Survivors vs. healthy volunteers, *p* = 0.007; survivors vs. nonsurvivors, *p* < 0.001. (c) Comparison of HRG in CAP patients grouped by days of hospitalization (0-7 days, 8-14 days, 15-30 days, and ≥31 days). Intergroup comparison, *p* = 0.121. (d) Comparison of HRG in CAP patients for different etiologies: bacteria, virus, atypical pathogen (including *Mycoplasma pneumoniae*, *Chlamydia pneumoniae*, and *Legionella pneumophila*), mixed pathogen, and unknown pathogen. Intergroup comparison, *p* = 0.101.

**Figure 2:** HRG levels are significantly negatively correlated with IL-6, CURB-65, PSI, and APACHE II. Abbreviations: APACHE: acute physiology, and chronic health evaluation; CURB-65: confusion, urea, respiratory rate, blood pressure, and age ≥ 65 years old; HRG: histidine-rich glycoprotein; IL-6: interleukin-6; PSI: pneumonia severity index.

**Figure 3:** Receiver operating curve (ROC) analysis of various parameters for prediction of 30-day mortality in patients with community-acquired pneumonia.

**Figure 4:** Cox survival analysis of 30-day cumulative survival in patients with community-acquired pneumonia. Analysis was stratified by HRG levels, as clinical parameters (age, bilateral lung infection, PCT, CURB-65, PSI, and APACHE II) were controlled. Abbreviations: APACHE: acute physiology and chronic health evaluation; CURB-65: confusion, urea, respiratory rate, blood pressure, and age ≥ 65 years old; HRG: histidine-rich glycoprotein; PCT: procalcitonin; PSI: pneumonia severity index.

**Table 1:** Baseline characteristics of the 160 patients with CAP on admission.

Parameters	Values		*p* value
	Survivors (*n* = 147)	Nonsurvivors (*n* = 13)	
Age (years)^a^	54 (35-67)	69 (56-77)	0.010
Age ≥ 65^b^	44 (29.9%)	7 (53.8%)	0.117
Males^b^	98 (66.7%)	7 (53.8%)	0.372
Comorbidities^b^			
Chronic heart failure	14 (9.5%)	2 (15.4%)	0.646
Diabetes mellitus	31 (21.1%)	4 (3.1%)	0.484
Cerebrovascular disease	28 (19.0%)	2 (15.4%)	0.999
Chronic liver disease	5 (3.4%)	2 (15.4%)	0.102
COPD	41 (27.9%)	7 (53.8%)	0.062
Active smokers^b^	78 (53.1%)	4 (30.8%)	0.153
Antibiotic pretreatment^b^	62 (42.2%)	2 (15.4%)	0.077
Laboratory results^a^			
WBC (×109/L)	8.4 (5.7-13.2)	12.7 (7.2-18.1)	0.074
CRP (mg/L)	76.0 (19.7-137.8)	95.0 (11.5-170.4)	0.694
PCT (*μ*g/L)	0.3 (0.1-2.2)	2.9 (0.3-9.4)	0.012
Interleukin-6 (pg/mL)	53.5 (18.4-98.1)	162.8 (101.3-735.8)	<0.001
Chest X-ray^b^			
Bilateral lung infection	87 (59.2%)	12 (92.3%)	0.018
Pleural effusion	21 (14.3%)	4 (30.8%)	0.124
CURB-65 score^a^	1 (0-2)	2 (2-3)	<0.001
PSI^a^	66 (44-95)	133 (118-148)	<0.001
APACHE II^a^	7 (4-11)	16 (14-19)	<0.001
Pathogen established^b^			
Bacteria	38 (25.9%)	3 (2.0%)	0.999
Virus	16 (10.9%)	0	0.366
Atypical pathogen	15 (10.2%)	0	0.613
Mixed pathogen	12 (8.2%)	0	0.601
Unknown	66 (44.9%)	10 (76.9%)	0.040

Abbreviations: APACHE: acute physiology and chronic health evaluation; CAP: community-acquired pneumonia; COPD: chronic obstructive pulmonary disease; CRP: C-reactive protein; CURB-65: confusion, urea, respiratory rate, blood pressure, and age ≥ 65 years old; PCT: procalcitonin; PSI: pneumonia severity index; WBC: white blood cell. ^a^Values are shown as a median (interquartile range). ^b^These parameters are shown as numbers (percentage).

**Table 2:** AUC and threshold for predicting 30-day mortality in patients with CAP based on different parameters.

Parameter	Threshold	Sensitivity (%)	Specificity (%)	AUC	*p* value	95% CI	
						Lower limit	Higher limit
Age (years)	>61	72.70	63.90	0.698	0.003	0.620	0.768
Bilateral lung infection	Bilateral	90.91	40.82	0.659	0.027	0.579	0.732
PCT (*μ*g/L)	>2.91	63.64	80.27	0.705	0.020	0.627	0.775
IL-6 (pg/mL)	>79.69	90.91	70.07	0.842	< 0.001	0.776	0.895
CURB-65	> 1	72.73	74.83	0.813	< 0.001	0.743	0.870
PSI	> 103	90.91	78.91	0.874	< 0.001	0.811	0.921
APACHE II	> 11	100	78.23	0.923	< 0.001	0.869	0.959
HRG (*μ*g/mL)	≤ 16.92	100	72.79	0.810	< 0.001	0.740	0.868

Abbreviations: APACHE: acute physiology and chronic health evaluation; AUC: area under the curve; CAP: community-acquired pneumonia; CI: confidence interval; CURB-65: confusion, urea, respiratory rate, blood pressure, and age ≥ 65 years old; HRG: histidine-rich glycoprotein; IL-6: interleukin-6; PCT: procalcitonin; PSI: pneumonia severity index.

**Table 3:** Cox proportional hazard regression analysis of the effects of multiple variables on 30-day survival of patients with CAP.

Variables	Univariate analysis		Multivariate analysis	
	HR (95% CI)	*p* value	HR (95% CI)	*p* value
Age	1.040 (1.000–1.082)	0.048		
Bilateral lung infection	4.387 (0.557–34.567)	0.160		
PCT (*μ*g/L)	1.033 (1.001–1.066)	0.046		
IL-6 (pg/mL)	1.000 (1.000–1.000)	0.001	1.001 (1.000–1.001)	0.001
CURB-65	1.864 (1.198–2.900)	0.006		
PSI	1.029 (1.011–1.047)	0.002		
APACHE II	1.397 (1.204–1.622)	< 0.001	2.020 (1.338–3.048)	0.001
HRG (*μ*g/mL)	0.949 (0.900–0.999)	0.047	0.889 (0.791–0.999)	0.049

Abbreviations: APACHE: acute physiology and chronic health evaluation; CAP: community-acquired pneumonia; CI: confidence interval; CURB-65: confusion, urea, respiratory rate, blood pressure, and age ≥ 65 years old; HR: hazard ratio; HRG: histidine-rich glycoprotein; IL-6: interleukin-6; PCT: procalcitonin; PSI: pneumonia severity index.

## Data Availability

The datasets generated and analyzed during the current study are not publicly available due to health privacy concerns, but are available from the corresponding author on reasonable request.
